The article "Management Strategy of Alzheimer's Patients under the Medical-Care Integration Model Based on Big Data Evaluation" was retracted in 2023. Reasons: signs of a paper mill; suspected computer-generated content; unreliable results or conclusions; concerns about the data.

# Management Strategy of Alzheimer's Patients under the Medical-Care Integration Model Based on Big Data Evaluation

**DOI:** 10.1155/2022/9896935

**Published:** 2022-10-11

**Authors:** Wei Sun, Jinxia Liu, Lihua Liu, Xiuzhi Wang

**Affiliations:** ^1^Baicheng Medical College, Baicheng, 137000 Jilin Province, China; ^2^School of Nursing, Capital Medical University, Beijing 100069, China; ^3^Beijing Huilongguan Hospital, Beijing 100096, China; ^4^Affiliated Hospital of Yanbian University, Yanji, 133000 Jilin Province, China

## Abstract

In the context of the era of big data, the management of Alzheimer's patients has aroused widespread concern in the society. What should the elderly and people with dementia do and how the society should accommodate these special groups have aroused heated discussions in the society. The goal of the medical-nursing integration model is to realize the integrated model of medical care-nursing-rehabilitation-old care, and to better satisfy the needs by providing medical services, rehabilitation care, and health management. The medical needs of the elderly can help the elderly maintain a healthy state; the elderly care needs can be better met through elderly care services, and the burden on families and society can be reduced. With the advancement of the medical-care integration model, new solutions have been provided for the management of senile dementia patients. Therefore, under the medical-care integration model, this paper managed Alzheimer's patients based on the big data algorithm based on association rules and compared it with the management of Alzheimer's patients under the traditional model, and drew the following conclusions: compared with the management satisfaction of Alzheimer's patients under the traditional model, family members and patients' total satisfaction with nursing management under the medical-care integration model was greatly improved; compared with the management of Alzheimer's patients under the traditional model, the incidence of adverse events in the management of Alzheimer's patients under the medical-care integration model was greatly reduced, which was reduced to 17.6%; under the medical-care integration model, the anxiety and depression scores of the elderly patients with dementia decreased rapidly; under the medical-care integration model, the living ability of senile dementia patients has been greatly improved; the use of the medical-care integration model to manage senile dementia patients has greatly improved the sleep quality, mental quality, and quality of life of senile dementia patients.

## 1. Introduction

In the traditional mode, the management of Alzheimer's patients is mainly managed by the family members of the patients. In this mode, doctors cannot grasp the physical conditions of Alzheimer's patients and doctors' return visits cannot be realistic, as well as patients' conditions and physical conditions cannot be adjusted in a targeted manner, which has caused huge social problems. On the one hand, the management of senile dementia patients is not standardized; on the other hand, family conflicts often arise due to the limitations of family management. Based on the above situations, it is urgent to improve the management system of senile dementia patients and propose new solutions for the management of senile dementia patients.

Alzheimer's disease patients, also known as Alzheimer's patients, often appear in the elderly group, and this issue has caused profound reflection in the society. Oskouei et al. focused on Alzheimer's patients and the care of their families using IoT-provided facilities to remotely monitor the behavior and health of these patients to reduce additional costs and respond to these patients in a timely manner [1]. Fiford et al. examined how longitudinal atrophy patterns in Mild Cognitive Impairment (MCI) and Alzheimer's disease change with age. Younger Alzheimer's patients have significantly faster rates of atrophy in the parietal and upper temporal lobes in bilateral forward flexion and ups and downs [2]. Naharci et al. reviewed the association between acetylcholinesterase inhibitors and osteoporotic fractures in Alzheimer's patients [3]. The purpose of Jasemin et al. is to organize the ability of attention and self-limitation in patients with Alzheimer's disease (AD), and organized 90 elderly people to participate in the experiment. It was concluded that total body position reeducation therapy had a significant effect on group differences in all outcomes [4]. Dominici et al. compared plasma *β*2-microglobulin serum levels in healthy subjects and subjects with dementia or cognitive impairment. *β*2-microglobulin serum may play a role in AD [5]. Ding et al. studied the biological function of Protein Phosphatase 2 AC (PP2AC) in the brain, and examined its spatiotemporal expression in mice and Alzheimer's patient brains and its involvement in neurological diseases. The findings revealed a spatiotemporally specific expression profile of PP2AC in the mouse brain, suggesting its biological significance. Its expression in the frontal cortex of patients with Alzheimer's disease is reduced, implying that PP2AC plays a potential role in the pathogenesis of Alzheimer's disease [6]. Merlo et al. proposed an approach that focuses on Alzheimer's patients but is of extraordinary value to the quality of life of their caregivers—the Alzheimer's Cafe [7]. Based on the status quo that Alzheimer's patients are widely valued in their lives, it is a social need and a national need to conduct research on this group.

In the era of big data, the combination of medical technology and nursing homes for management brings more possibilities to the elderly, and the integration of medical and nursing care has also attracted the attention of scholars. Sivakumar et al. proposed a care plan for aged care that highlights the benefits of being proactive for mental health professionals to help families and service users address future care planning issues [8]. Pekkarinen et al. used the “loophole approach” to investigate innovation opportunities related to the digitization of healthcare and aged care services [9]. The Caic et al. study investigated the potential role of service robots (i.e., social assistance robots) in elderly care value networks [10]. Lian investigated the needs of elderly people in Guangxi for elderly care services. Combined with the development status of the elderly care service in Guangxi, three smart elderly care paths were proposed to adapt to the characteristics of regional development: community grid management+community elderly care security, smart home+home care, and the Internet+hospital medical care+home care [11]. Sg et al. assessed GPs' perceptions of what factors in long-term care reform facilitate and hinder the delivery of integrated person-centered care for older people in the Netherlands. Case studies were conducted through semi-structured interviews, using the Health Alliance (HALL) framework as a framework for thematic analysis, and recommendations were made. The use of a central location provides primary health and social services and integrates regional ICT structures to improve the exchange of patient information, and reduce fragmentation of home care [12]. Bovenkamp et al. drew on concepts from organizational research to show that the work of caregivers, healthcare managers, and external actors is often decoupled, and caregivers experience regulatory stress when the origin and function of rules are unclear [13]. Deep et al. reviewed and discussed current research trends in aged care, and their outcomes and implications for elderly care. In order to help them live in a safer environment, the increasing cost of nursing care and the shortage of health care personnel have prompted the recent demand for home-based assisted living [14]. At this stage, no research has been found to analyze the management of Alzheimer's patients under the medical-care integration mode. Therefore, this paper analyzed the management of Alzheimer's patients under the medical-care integration mode.

In order to give more care to Alzheimer's patients and promote the harmonious development of society, this paper used a big data algorithm based on association rules to manage the Alzheimer's patients under the integration of medical care and health care, and compared it with the management of Alzheimer's patients under the traditional model. The relevant content was investigated, and the feasibility conclusion was drawn. This article provides a new solution for the management of Alzheimer's patients, so as to ease family conflicts.

## 2. Big Data Algorithm Based on Association Rules

### 2.1. Establishment and adjustment of association rules

Apriori algorithm is one of the most widely used algorithms in association rules, and it is used to analyze big data of patient diagnosis [15]. The algorithm needs to search for frequent itemsets in patient diagnostic big data, and generate association rules to determine the relationship between itemsets in patient diagnostic big data. The specific process is as follows.

The confidence level is set to represent the probability that itemsets A and B occur at the same time in the patient diagnosis big data, and then there are

(1) $$\begin{array}{c} \text{Support}\left(A\Rightarrow B\right)=P\left(A\cup B\right)=\frac{\text{Support}\_\text{count}\left(A\cup B\right)}{\text{Total}\_\text{count}}. \end{array}$$

Confidence is used to establish association rules, which can be expressed by

(2) $$\begin{array}{c} \text{Confidence}\left(A\Rightarrow B\right)=P\left(B\left|A\right.\right)=\frac{\text{Support}\_\text{count}\left(A\cup B\right)}{\text{Support}\_\text{count}\left(A\right)}. \end{array}$$

The Apriori algorithm is used to calculate the support degree to determine the frequent itemsets of the patient diagnosis big data, and the frequent itemsets are used to generate strong association rules to realize the analysis of the patient diagnosis big data. The association between the data of this algorithm is weak, so the association rules need to be adjusted in the Apriori algorithm [16].

It is assumed that *a*_*ik*_ represents the attribute *x*_*j*_ of the *k* patient diagnosis big data, and *μ*_*ai*_ and *σ*_*ai*_ represent the mean and standard deviation of the patient diagnosis big data set, respectively, and *γ*_min_ represents the minimum confidence degree. The calculation formulas can be expressed as

(3) $$\begin{array}{c} \mu_{ai}\left(T\right)=\frac{\sum_{k\in T}\left(a_{ik}\right)}{\left|T\right|},\\ a_{ai}\left(T\right)=\sqrt{\frac{\sum {\left(a_{ik}-\mu_{ai}\left(T\right)\right)}^{2}}{\left|T\right|}},\\ \gamma_{\min}=\mu_{ai}\left(T_{j}\right)-\mu_{ai}\left(T-T_{j}\right). \end{array}$$

After adjusting the association rules, a new association rule is obtained

(4) $$\begin{array}{c} \text{Confidence}\left(A\Rightarrow B\right)=\frac{\mu_{ai}\left(T_{x_{j}}\right)-\mu \left(T-T_{x_{j}}\right)}{\sigma_{a_{i}}\left(T_{x_{j}}\right)/\sqrt{\left|T_{x}\right|}}. \end{array}$$

### 2.2. Data attribute reduction of genetic algorithm

In the process of data mining by association rules, the genetic algorithm is introduced to represent the feasible solutions of the problem as chromosomes. The fitness function is established to determine the optimal solution of the problem, and the genetic algorithm is used to reduce the data attributes [17].

It is assumed that the Apriori algorithm and the FP-Growth algorithm are used to extract the big data of patient diagnosis, and the obtained solution is

(5) $$\begin{array}{c} x=\left(x_{1},x_{2},\cdots ,x_{n}\right). \end{array}$$

The assumptions are

(6) $$\begin{array}{c} Z=\left\{X_{i}\right.=\left(x_{i1},x_{i2},\cdots ,x_{\text{in}}\right),\left.i=1,2,\cdots ,n\right\}. \end{array}$$

In the formula, *Z* represents a general group of patients with diagnostic big data attributes, *X*_*i*_ represents the chromosome individual in the population, and *x*_*i*_ represents the gene in the chromosome.

If the solution corresponding to chromosome individual *X* is *x*, then the fitness of individual *X* is:

(7) $$\begin{array}{c} \text{Fit}\left(X\right)=\left\{\begin{array}{c} -C_{\min}+f\left(x\right),\\ 0, \end{array}\right.\begin{array}{c} f\left(x\right)>C_{\min}\\ \text{otherwise} \end{array}, \end{array}$$

or:

(8) $$\begin{array}{c} Fit\left(X\right)=\frac{1}{C_{\min}-f\left(x\right)}. \end{array}$$

The minimum value of the objective function *f*(*x*) is calculated. According to the above, the fitness of the individual *X* can be expressed as:

(9) $$\begin{array}{c} \text{Fit}\left(X\right)=\left\{\begin{array}{c} C_{\min}-f\left(x\right),\\ 0, \end{array}\right.\begin{array}{c} f\left(x\right)<C_{\min}\\ \text{otherwise} \end{array}, \end{array}$$

or:

(10) $$\begin{array}{c} \text{Fit}\left(X\right)=\frac{1}{-C_{\min}+f\left(x\right)}. \end{array}$$

The probability *P*(*x*_*i*_) that any individual *x*_*i*_ of the population is selected and inherited to the next generation can be expressed as

(11) $$\begin{array}{c} P\left(x_{i}\right)=\frac{\text{Fit}\left(x_{i}\right)}{\sum_{j=1}^{n}\text{F}\text{it}\left(x_{j}\right)}. \end{array}$$

In the formula, Fit(*x*_*i*_) represents the adaptability of *x*_*i*_.

### 2.3. Big data mining of patient diagnosis based on decision tree algorithm

The information entropy corresponding to the dataset *S* can be expressed as

(12) $$\begin{array}{c} I\left(s_{1},s_{2},\cdots ,s_{n}\right)=-\overset{\text{m}}{\underset{\text{i}=1}{\sum }}P_{\text{i}}\log_{2}\left(P_{i}\right). \end{array}$$

The information entropy of attribute *A* divided samples is

(13) $$\begin{array}{c} E\left(A\right)=\overset{v}{\underset{j=1}{\sum }}\frac{s_{1j}+\cdots +s_{nj}}{s}I\left(s_{1j},\cdots ,s_{mj}\right). \end{array}$$

For a given subset *S*_*j*_, the expected information can be calculated by

(14) $$\begin{array}{c} I\left(s_{1j},\cdots ,s_{mj}\right)=-\overset{m}{\underset{i=1}{\sum }}p_{ij}\log_{2}\left(p_{ij}\right). \end{array}$$

According to the calculated information entropy and expected information, the information gain obtained by dividing the sample set *S* by attribute *A* is

(15) $$\begin{array}{c} \text{Gain}\left(A\right)=I\left(s_{1j},\cdots ,s_{mj}\right)-E\left(A\right). \end{array}$$

By optimizing the classification attributes, the initial amount of information corresponding to attribute *A* is obtained as

(16) $$\begin{array}{c} S\text{plit In }f_{A}\left(A\right)=-\overset{v}{\underset{j=1}{\sum }}\frac{\left|S_{j}\right|}{S}\times \log_{2}\left(\frac{\left|S_{j}\right|}{S}\right). \end{array}$$

The formula for calculating the information gain rate is

(17) $$\begin{array}{c} \text{Gain Ratio}\left(A\right)=\frac{\text{Gain}\left(A\right)}{\text{Split In }f_{A}\left(A\right)}. \end{array}$$

The established decision tree mining model can be expressed as

(18) $$\begin{array}{c} \psi =\overset{v}{\underset{j=1}{\sum }}\frac{s_{1j}+\cdots +s_{mj}}{s}•\text{Gain Ratio}\left(A\right). \end{array}$$

## 3. Evaluation of Management Strategies for Elderly Patients with Dementia

### 3.1. Management of Alzheimer's patients under the traditional model

Under the traditional model, most Alzheimer's patients are cared for by family members in their own homes [18]. When their family members find out that there is a problem with the patient, they would contact the hospital and send the patient to the hospital, so as to realize the management of Alzheimer's patients. Under this model, there are great drawbacks. Family members cannot grasp the patient's physical condition, nor can they give timely feedback to the doctor on the patient's physical condition, which greatly reduces the efficiency of patient treatment. This situation can be seen in Figure 1.

In the traditional model, the management of patients with Alzheimer's mainly relies on the family members of the patients, because the patients with dementia cannot receive the information conveyed by their family members, and there is a great communication barrier between the two. As a result, conflicts often arise between patients and their families, resulting in family crises. In this stalemate, patients and their families cannot express their love for each other and cannot build a harmonious family relationship.

### 3.2. Follow-up management of patients with dementia

Now the hospital has also implemented follow-up management for the management of senile dementia patients [19]. This management method requires doctors to understand the basic situation of the patient and give targeted guidance to the caregivers, but the management method is not yet mature, and there are still major problems: the quality of follow-up management is not high and the follow-up plan is not comprehensive enough, as well as the information construction of follow-up management is insufficient. Based on this, this management method is not suitable for most families of Alzheimer's patients. The specific problem can be seen in Figure 2.

Based on the problems existing in the implementation of the follow-up management system, there are also corresponding management methods, such as strengthening the management of the service attitude of the follow-up personnel and training them, as well as setting up a special follow-up service quality evaluation system, and prompting them to consciously improve the service quality. A comprehensive platform for Alzheimer's patients is established to manage the Alzheimer's patients in a unified manner, and the patient's physical condition data is updated in real time, thereby improving the scientific nature of caring for Alzheimer's patients. This management method is feasible, but in the traditional family management model, it is extremely difficult to turn the ideal into reality. Therefore, it is necessary to consider practical factors and propose new solutions for the management of Alzheimer's patients.

### 3.3. Management of Alzheimer's patients under the medical-care integration model

Under the medical-care integration model, medical institutions are transformed into rehabilitation institutions or nursing homes that provide integrated medical and elderly care services [20]. Because hospitals and nursing homes are linked together, they can provide more scientific guidance to patients. Nursing homes also have the function of hospitals, and the management of Alzheimer's patients is more humane. The institution is not only equipped with complete medical facilities but also with professional management personnel, which can not only realize real-time monitoring of the physical data of Alzheimer's patients but also timely treat them. The specific content can be seen in Figure 3.

The nursing home has the functions of a hospital and a nursing home. It not only provides a comfortable living environment for Alzheimer's patients but also is equipped with a professional nursing team, whose members include not only doctors, nurses but also nurses. Hospitals and elderly care service institutions have opened green channels. Professional medical personnel from hospitals regularly visit elderly care institutions for inspections. Health data and elderly information are exchanged, so that they can grasp the physical data of patients in a timely manner, and give good medical advice to prevent the deterioration of patients' conditions.

## 4. Evaluation of Management Strategies for Alzheimer's Patients under the Mode of Medical and Nursing Integration

In order to analyze the management strategy of senile dementia patients under the medical and nursing integration model, 40 senile dementia patients were selected in a certain hospital and divided into two groups. Among them, the control group is managed according to the traditional model, which is recorded as Group A; the experimental group adopted the medical and nursing integration model to manage the Alzheimer's patients, which is recorded as Group B. The patients are managed in groups based on different management modes, and the test data is recorded and analyzed.

### 4.1. Comparison of baseline data between the two groups

Group A and Group B had 20 cases each. Group A was 64 to 76 years old, with an average age of (65.1 ± 6.4) years, height of (154.3 ± 4.6) cm, weight of (52.3 ± 4.1) kg, and disease duration of (2.5 ± 1.2) years; Group B was 54 to 65 years old, with an average age of (60.2 ± 5.6) years, height (156.1 ± 4.3) cm, weight (53.4 ± 3.5) kg, and disease duration (3.1 ± 0.6) years. The difference between the two is reflected in the slight difference in the course of disease, and the disease course of the patients in the experimental group is longer than that of the patients in the control group. The specific results can be seen in Table 1:

### 4.2. Survey on the overall satisfaction rate of patients and their families on nursing management

Patients and their families' satisfaction with nursing management can reflect the advantages and disadvantages of the management model, so that they can be improved in a targeted manner. In order to investigate whether the management of senile dementia patients under the medical-care integration model meets the daily needs of the patients and whether it is truly for the sake of the patients, this paper records the satisfaction of the patients and their families in Groups A and B in Figure 4.

As can be seen from Figure 4, compared with Group A, the satisfaction of the family members of patients in Group B with nursing management increased by 25%, and the satisfaction with nursing management of patients in Group B increased by 30%. Based on this, it can be seen that patients and their families have greatly improved the overall satisfaction with nursing management under the medical-nursing integration model. According to the interview, more family members of patients were more willing to accept and try the management of Alzheimer's patients under the integrated medical care model. The main reasons are in this mode, the nursing staff gives the patient more company and the medical staff is in place in time when the symptoms of the elderly occur, as well as the elderly no longer feel lonely under the care of the nursing staff. The elderly also get rid of the trouble of being unaccompanied, and the nursing staff also timely feedback the patient's physical condition to the patient's family member. Family members can also grasp the changes in the patient's physical state in time, which also implicitly promotes the feelings of patients and their families.

### 4.3. Investigation on the incidence of adverse events

Adverse events mainly refer to pressure ulcers, falling from bed, falls, aspiration, scalding, and other events that senile dementia patients may encounter in the process of receiving care, which may have adverse effects on the body and mind of the elderly. The occurrence of adverse events may reflect the attentiveness of the nursing staff to the patient, and can indicate whether the nursing staff is attentive to the patient. The occurrence of adverse events in Groups A and B within one month was recorded in Figure 5.

As can be seen from Figure 5, within one month, there were 2 pressure ulcers, 5 falls from bed, 4 falls, 0 aspiration, and 3 scalds within one month, with an overall incidence rate of 82.4%; in the medical-care integration mode, there were 0 pressure ulcers, 2 falls from bed, 1 fall, 0 aspiration, and 0 scald, with a total incidence rate of 17.6%. It can be seen that the incidence of adverse events in the management of Alzheimer's patients under the medical and nursing integration model is significantly lower than that in the traditional mode. Among them, there were 0 incidents of pressure ulcers, aspiration incidents, and scalding incidents, indicating that the nursing staff provided strong care for the patients and prevented the occurrence of harmful incidents. Based on this, family members are more willing to send Alzheimer's patients to nursing homes. Professional care of patients can prevent patients from suffering from adverse events such as pressure ulcers, falls from bed, falls, aspiration, and scalding.

### 4.4. Anxiety and depression score survey of patients

Many Alzheimer's patients often suffer from anxiety and depression when they are suffering from illness, and they are in a state of lack of energy for a long time, which would aggravate the patient's condition and bring adverse effects to the patient in the long run. The score test of patients' anxiety and depression can reflect the mood changes of patients, and can reflect the management attitude and quality of managers from the side, so as to conduct targeted management evaluation of patients. Based on this, the anxiety and depression scores of patients in Group A and Group B within one year were recorded in Figure 6:

It can be seen from Figure 6 that the anxiety and depression scores of the patients in Group A and Group B decreased month by month within one year, and the patients' anxiety and depression scores decreased faster in the management of Alzheimer's patients under the medical-care integration model. Patients' anxiety and depression scores at the end of the month were lower than those of Alzheimer's patients in the traditional model. The reason is that the nursing staffs put their hearts and minds in the process of caring for the Alzheimer's patients and regard the patients as their relatives, and take the trouble to communicate and serve them to help patients with practical actions and alleviate the suffering of patients. It can be seen that under the medical-nursing integration model, the anxiety and depression scores of Alzheimer's patients decreased rapidly, and the management of nursing staff played a role in regulating the patients' emotions.

### 4.5. Patient living ability score survey

Alzheimer's patients often suffer from forgetfulness and inability to take care of themselves. They cannot handle communication, activities, and family life by themselves. Therefore, the investigation of the living ability of senile dementia patients can reflect the quality of the management mode. The patient's living ability can be divided into mental function, organ function, communication, activity, self-care, family life, economic, and social life, with a full score of 100 points. Among them, 15 points for mental function, 15 points for organ function, 20 points for communication, 10 points for activities, 10 points for self-care, 20 points for family life, and 10 points for economic and social life. The living ability level of Group A and Group B was investigated, and the results were recorded in Figure 7.

As can be seen from Figure 7, the mental function score of Group A patients was 9.1 points, the organ function score was 12.5 points, the communication score was 13.5 points, the activity score was 6.5 points, the self-care score was 14.6 points, the family life score was 2.3 points, and the economic and social life score was 6.4 points; in Group B, the score of mental function was 10.6, the score of organ function was 14.4, the score of communication was 15.8, the score of activity was 8.8, the score of self-care was 17.2, the score of family life was 9.4, and the score of economic and social life was 8.1. Therefore, under the medical-care integration model, the living ability of Alzheimer's patients has been greatly improved. Among them, the improvement in family life is the fastest, which shows that the family life of the patients is not blocked under the medical and nursing integration model.

### 4.6. Investigation on sleep quality, mental quality, and quality of life of patients

Alzheimer's patients often suffer from poor sleep quality, weak mental quality, and poor quality of life due to lack of careful care. In order to improve the sleep quality and quality of life of patients, this paper uses the form of scoring to score the sleep quality and quality of life of Alzheimer's patients under the medical-care integration model, and compares it with the scores of sleep quality, mental quality and quality of life of Alzheimer's patients in the traditional mode. Group A represents the scores of sleep quality, mental quality, and quality of life of Alzheimer's patients under the traditional model, and Group B represents the sleep quality, mental quality, and quality of life scores of Alzheimer's patients under the medical-care integration model. The sleep quality of patients is evaluated by the sleep quality index PSQI and the quality of life is evaluated by ADL. It is known that the lower the PSQI score, the higher the patient's mental quality; the higher the ADL score, the higher the patient's quality of life. The survey results are recorded in Figure 8.

According to Figure 8, compared with Group A, the Pittsburgh Sleep Quality Index (PSQI) value of the patients in Group B was decreased; that is, the sleep quality of the patients was improved; the Activities of Daily Living (ADL) value of the patients in the Group B was increased; that is, the quality of life of the patients was improved. To sum up, the use of the medical-care integration model to manage Alzheimer's patients has greatly improved the sleep quality, mental quality, and quality of life of Alzheimer's patients. Therefore, it is beneficial to manage senile dementia patients in the mode of medical and nursing integration.

## 5. Conclusion

In this paper, the big data algorithm based on association rules conducted a survey on Alzheimer's patients in the medical and nursing integration mode, and compared it with the patient management in the traditional mode. The conclusion is that the overall satisfaction rate of patients and their families on nursing management has increased and the incidence of adverse events has decreased, as well as the patient's anxiety and depression score has been reduced month by month. The patient's living ability score has greatly improved, and the patient's sleep quality, mental quality, and quality of life have improved. Therefore, the management of Alzheimer's patients is more standardized and scientific under the medical and nursing integration model, which can not only improve the patient's ability but also promote the harmonious development of the family.

## Figures and Tables

**Figure 1:** Disadvantages of the traditional model of managing patients with dementia.

**Figure 2:** Disadvantages of follow-up management of Alzheimer's patients.

**Figure 3:** Management of Alzheimer's patients in the medical care integration model.

**Figure 4:** Overall satisfaction rate of patients and their families with nursing management.

**Figure 5:** Incidence of adverse events.

**Figure 6:** Survey of patient anxiety and depression scores.

**Figure 7:** Patient living ability score survey.

**Figure 8:** Survey on sleep quality, mental quality and quality of life of patients.

**Table 1:** Comparison of baseline data between the two groups.

Project	A group (*n* = 20)	B group (*n* = 20)
Age (years)	65.1 ± 6.4	60.2 ± 5.6
Height (cm)	154.3 ± 4.6	156.1 ± 4.3
Weight (kg)	52.3 ± 4.1	53.4 ± 3.5
Disease duration (years)	2.5 ± 1.2	3.1 ± 0.6

## Data Availability

The data of this paper can be obtained through the email to the authors.
